The article "Punicalagin Alleviates Aged Bronchial Asthma by Inhibiting Th2 Differentiation through IL-4/STAT6 and Jagged1/Notch Pathways" was retracted in 2023. Reasons: signs of a paper mill; suspected computer-generated content; unreliable results or conclusions; lack of ethics approval or compliance.

# Punicalagin Alleviates Aged Bronchial Asthma by Inhibiting Th2 Differentiation through IL-4/STAT6 and Jagged1/Notch Pathways

**DOI:** 10.1155/2022/1184677

**Published:** 2022-01-30

**Authors:** Li Yu, Jianying Li

**Affiliations:** The Division of General Medicine, The People's Hospital of Guangxi Zhuang Autonomous Region, Nanning 530021, Guangxi Zhuang Autonomous Region, China

## Abstract

**Objective:**

To explore the therapeutic effect and mechanism of punicalagin on bronchial asthma in the elderly.

**Methods:**

Peripheral venous blood was collected from healthy people and elderly patients with bronchial asthma. Peripheral blood mononuclear cells (PBMCs) were isolated and cultured. PBMCs in the patient group were treated with different concentrations (0, 50, 100, and 200 mg/L) of punicalagin (PUN). MTT assay was used to detect cell activity, ELISA was used to detect the levels of IFN-*γ*, IL-2, IL-4, and IL-5, and Western blotting was used to detect the protein levels of p-STAT6, Jagged1, and GATA3.

**Result:**

MTT results showed that 50–200 mg/L PUN had no cytotoxicity to PBMCs within 24 h. ELISA results showed that the levels of IFN-*γ* and IL-2 in the serum of the patients were significantly lower than those of healthy people, and the levels of IL-4 and IL-5 were significantly higher than those of the healthy people. PUN treatment significantly increased the levels of IFN-*γ* and IL-2 in the supernatant of PBMCs culture, while significantly decreased the levels of IL-4 and IL-5, and the change was proportional to the concentration of PUN. Western blotting results showed that the levels of p-STAT6, Jagged1, and GATA3 protein in PBMCs of patients were significantly higher than those of the healthy people. PUN treatment could significantly reduce the expression of p-STAT6, Jagged1, and GATA3 protein in PBMCs of patients, and the reduction level was proportional to PUN concentration.

**Conclusion:**

PUN can inhibit Th2 differentiation and regulate Th1/Th2 balance by regulating IL-4/STAT6 and Jagged1/Notch pathways to alleviate the progress of bronchial asthma in the elderly.

## 1. Introduction

Bronchial asthma, also known as asthma, is a chronic airway inflammation involving eosinophils, mast cells, lymphocytes, neutrophils, and other cells and various media, which is common to the elderly [1]. This chronic inflammation is associated with airway hyperresponsiveness, characterized by wheezing, chest tightness, shortness of breath and cough, and reversible episodes [2]. Due to the elderly patients with physical function is constantly weakening, immune ability is also declining, respiratory system vulnerable easily leads to respiratory tract infection, and then cause bronchial asthma, if not timely treated, will affect their health. Bronchial asthma is sudden, often occurs at night, prone to complications, severe and even lead to lung infection, and even respiratory failure to death. The global incidence of asthma has reached about 300 million, showing a rapid upward trend in China [3]. Bronchial asthma has no radical treatment at present. At the same time, due to the characteristics of acute onset, long course of disease, and easy recurrence, it is a difficult problem in respiratory-related diseases. In the pathogenesis, the imbalance of Th1/Th2 in CD4+ Th cell subsets is currently recognized as the immunological pathogenesis of asthma [4]. Studies have shown that patients with asthma have excessive differentiation of Th2 cells and excessive secretion of Th2 cytokines [5].

Punicalagin (PUN) is a polyphenolic active ingredient extracted from pomegranate plants [6]. In recent years, studies have found that PUN has strong antioxidation, antiproliferation, and tumor inhibition effects, as well as antiatherosclerosis and anti-inflammatory functions. In primary cultured chondrocytes, PUN can inhibit LPS-induced inflammatory response [7]. However, its specific mechanism of action has not been elucidated in depth. At present, there are few studies on the role of PUN in the development of bronchial asthma. Therefore, this study aims to explore the effect and mechanism of PUN on the process of bronchial asthma in the elderly and provide scientific data and basis for the treatment of bronchial asthma by PUN.

## 2. Materials and Methods

### 2.1. Participants

In this study, 30 elderly patients with bronchial asthma admitted to our hospital from March 2021 to November 2021 were selected as the observation group, and 30 healthy people in the same period were selected as the control group. General data such as age, gender, and BMI were not statistically different between the two groups and were comparable. This study has been approved by the hospital ethics committee. The inclusion criteria of patients are as follows: all patients met the diagnostic criteria of bronchial asthma, referring to the diagnostic criteria of the 1997 Guidelines for the Prevention and Treatment of Bronchial Asthma in China; course of disease greater than 6 months; age >65 years; and agreed to this clinical trial and signed the informed consent form. Exclusion criteria are as follows: with other immune or metabolic diseases; with other malignant tumors; with infectious or blood diseases; and refusing to accept this clinical trial.

### 2.2. Cell Culture

A total of 10 mL peripheral venous blood was collected from patients with bronchial asthma and healthy adults by sterile working. Heparin was used for anticoagulation. 5 mL of peripheral blood mononuclear cells (PBMCs) was separated by the Ficoll method. PBMCs were cultured in RPMI1640 medium containing 10% fetal bovine serum and cultured in a 5% CO_2_ incubator at 37°C.

### 2.3. Punicalagin Treatment

PBMCs from patients with bronchial asthma were taken, and the cell density was adjusted to 1 × 10^6^/mL, which was inoculated in 24-well plates. The cells in the control group were treated with PBS, and the cells in the experimental group were treated with low (50 mg/L), medium (100 mg/L), and high (200 mg/L) concentrations of PUN, respectively. Routine culture for 24 hours for subsequent experiments.

### 2.4. Cell Viability Assay

PBMCs were collected from each group, the culture medium was removed, washed once with PBS, 20 *μ*L of 0.5% MTT diluted with serum-free culture medium was added to each well, and cultured at 37°C for 4 h in a 5% CO_2_ incubator. The culture medium was discarded, and 150 *μ*L DMSO (Sigma-Aldrich) was added to each well to oscillate until complete dissolution. A microplate reader (Labsystems) was used to detect OD_570nm_ absorbance. Besides, the experiment was performed three times, independently.

### 2.5. Enzyme-Linked Immunosorbent Assay (ELISA)

The ELISA kit (eBioscience) was used to detect the levels of IFN-*γ*, IL-2, IL-4, and IL-5 in the serum of healthy people and patients and in the supernatant of PBMCs culture medium of patients. The operation was carried out in strict accordance with the instructions of the kit.

### 2.6. Western Blotting

The total protein of PBMCs were extracted by RIPA lysate, and the protein concentration was measured by the BCA protein detection kit (Beyotime Biotechnology). The protein was separated by SDS-PAGE electrophoresis, cut and transferred to PVDF membrane (Sigma), and blocked with 5% skim milk powder at room temperature for 4 h. Added protein primary antibodies including anti-STAT6 (ab32108), anti-Jagged1 (ab109536), and anti-STAT3 (ab199428) (Abcam) and incubated overnight at 4°C. The second antibody (Abcam) was added at room temperature the next day. After incubation for 1 h, the gel imaging system was exposed, and the gray value of the band was analyzed by Image-Pro Plus 6.0.

### 2.7. Statistical Analysis

Data used were expressed as mean ± SD. The differences were analyzed using Student's *t*-test or one-way analysis of variance. All statistical analyses were performed using SPSS 17.0 software and GraphPad Prism 8.0 software. A difference was considered statistically significant with *P* < 0.05.

## 3. Results

### 3.1. Effect of Punicalagin on Activity of PBMCs

Compared with the control group, each concentration of PUN had no significant effect on the activity of PBMCs, indicating that 50–200 mg/L PUN had no cytotoxicity to PBMCs within 24 h (Figure 1).

As shown in Figure 2, the serum levels of IFN-*γ* and IL-2 in asthma patients were significantly lower than those in healthy people (*P* < 0.05, Figure 2(a)), and the levels of IL-4 and IL-5 were significantly higher than those in healthy people (*P* < 0.05, Figure 2(b)). After PBMCs were treated with different concentrations of PUN, the levels of the above cytokines in the supernatant were detected. Compared with the control group, the levels of IFN-*γ* and IL-2 in the PUN treatment group were significantly increased (*P* < 0.05), and the levels of IL-4 and IL-5 were significantly decreased (*P* < 0.05). The degree of change was proportional to the concentration of PUN (Figures 2(c)–2(f)).

### 3.2. Effects of Punicalagin on p-STAT6, Jagged1, and GATA3 Protein Levels in PBMCs

As shown in Figure 3, after PBMCs were treated with different concentrations of PUN, compared with the control group, the expression levels of p-STAT6, Jagged1, and GATA3 in the PUN treatment group were significantly decreased (*P* < 0.05), which suggested that PUN significantly inhibited the expression of p-STAT6, Jagged1, and GATA3.

## 4. Discussion

Bronchial asthma is a chronic respiratory disease involving multiple cells and cellular components, which seriously affects people's physical and mental health [1]. The main manifestations are airway inflammation, airway hyperresponsiveness, and airway remodeling [2]. Elderly people because of physical decline and poor resistance are more prone to bronchial asthma. The pathogenesis of bronchial asthma is related to the regulation of multiple signaling pathways, and immune and inflammatory regulatory factors play an important role. During the treatment of asthma, some drugs can cause some adverse reactions, such as eye problems, gastric ulcer, elevated blood pressure, and poisoning [8]. Therefore, in recent years, the natural product development of safe and effective antiasthma drugs related research is also increasing.

PUN is a hydrolyzed tannin, which is the most important active ingredient in pomegranate peel polyphenols (about 60–70%). It can be isolated from a few plants such as pomegranate peel and leaves of euryale seed tree and Chebulae Fructus. Pomegranate peel is the dry peel of pomegranate, a traditional Chinese herbal medicine. PUN has a wide range of pharmacological effects, such as anti-inflammatory [9], antibacterial [10], antioxidant [11, 12], and antitumor [13].

Many studies have shown that the imbalance of Th1/Th2 functions and the dominant differentiation of Th2 cells may be one of the important mechanisms leading to asthma. The cytokine environment in which Th cells are located is the most intense regulatory factor of Th0 cells to differentiate into Th1 and Th2 [14]. IFN-*γ* and IL-2 are one of the two multifunctional factors in Th1 cytokines. IFN-*γ* is involved in the immune balance regulation system of Th1/Th2, and the higher the level is, the stronger the protective effect on the body is. IL-2 is one of the earliest discovered cytokines with a wide range of biological activities. It plays an important role in regulating the body's immune function and can effectively regulate the activity and value-added development of human T cells, natural killer cells, and monocytes. IL-4 and IL-5 are two representative factors in Th2 cytokines. Both of them can stimulate B cells to synthesize IgE and promote Th2 cells, while IL-4 also inhibits Th1. The role of cytokines requires intracellular signaling pathways and nuclear transcription factors. The existing data suggest that there are two groups of mutually antagonistic transcription factors in the differentiation of Th0, STAT6/STAT4, and T-bet/GATA3. IL-12 makes cells differentiate into Th1 through STAT4 and T-bet, while IL-4 makes cells differentiate into Th2 through STAT6 and GATA3 [15, 16]. Therefore, transcription factors play an important role in the differentiation of Th cells. In this study, the levels of cytokines in serum of healthy people and asthma patients were detected. It was found that the levels of IFN-*γ* and IL-2 in serum of asthma patients were significantly lower than those of healthy people, and the levels of IL-4 and IL-5 were significantly higher than those of healthy people. Then, PBMCs were treated with PUN. The results showed that the levels of IFN-*γ* and IL-2 in the culture supernatant were significantly increased, and the levels of IL-4 and IL-5 were significantly decreased. Western blotting results showed that the expression of p-STAT6 and GATA3 in PBMCs was significantly decreased. Therefore, it is speculated that PUN can inhibit Th2 differentiation and regulate Th1/Th2 balance through IL-4/STAT6.

The Notch pathway is an evolutionary highly conserved signaling pathway, which is composed of Notch receptors, Notch ligands, cell effectors, effectors, and their regulators. The Notch pathway plays a wide regulatory role in human body, such as promoting cell differentiation, stem cell proliferation, cell movement, and cycle [17–19]. As far as the respiratory system is concerned, the change of the Notch pathway plays an important role in lung diseases such as asthma, COPD, pulmonary hypertension, and lung cancer. Many studies have shown that the Notch signaling pathway and T lymphocyte regulation are jointly involved in the occurrence and development of asthma [20–22]. Among them, Notch ligand Jagged is the main factor affecting Th2 differentiation [23]. GATA3 is an important transcription factor of the development of Th2 cells, which is essential for Notch-mediated Th2 cell differentiation. The deletion of GATA3 can transform Notch from the inducer of Th2 to the inducer of Th1 differentiation. Notch and Jagged ligands induced GATA3 elevation and induced CD4+ *T* to differentiate into Th2 cells [24, 25]. The results of this study showed that the protein levels of Jagged1 and GATA3 in PBMCs were significantly decreased after PUN treatment, so it was speculated that PUN could inhibit Th2 differentiation through the Jagged1/Notch pathway.

In summary, PUN can inhibit Th2 differentiation by regulating IL-4/STAT6 and Jagged1/Notch pathways to regulate Th1/Th2 balance, thereby alleviating the progression of bronchial asthma in the elderly.

It can provide theoretical basis for the development of new drugs for the treatment of bronchial asthma in the elderly. However, this study has certain limitations, and subsequent in vivo experiments are still needed to explore the effect of PUN on bronchial asthma in the elderly.

## Figures and Tables

**Figure 1:** Effect of punicalagin on viability of PBMCs (^*∗*^*P* < 0.05). Effect of punicalagin on levels of cytokines in PBMCs.

**Figure 2:** Effect of punicalagin on IFN-*γ*, IL-2, IL-4, and IL-5 expression in PBMCs (^*∗*^*P* < 0.05, ^*∗∗*^*P* < 0.01). (a, b) Serum IFN-*γ*, IL-2, IL-4, and IL-5 levels in healthy people and patients with asthma. (c) Effects of different concentrations of PUN on IFN-*γ* levels. (d) Effects of different concentrations of PUN on IL-2 levels. (e) Effects of different concentrations of PUN on IL-4 levels. (f) Effects of different concentrations of PUN on IL-5 levels.

**Figure 3:** Effect of PUN on p-STAT6, Jagged1, and GATA3 protein expression in PBMCs (^*∗*^*P* < 0.05, ^*∗∗*^*P* < 0.01). (a) Western blotting results. (b) Effects of different concentrations of PUN on the expression level of p-STAT6 protein. (c) Effects of different concentrations of PUN on the expression level of Jagged1 protein. (d) Effects of different concentrations of PUN on the expression level of GATA3 protein.

## Data Availability

The data used to support the findings of this study are available from the corresponding author upon request.
